The article "Analysis of the Role of Continuous Early Intervention in Improving the Quality of Life of Breast Cancer Patients" was published in 2022. Journal: Comput Intell Neurosci.

# Analysis of the Role of Continuous Early Intervention in Improving the Quality of Life of Breast Cancer Patients

**DOI:** 10.1155/2022/3054587

**Published:** 2022-06-16

**Authors:** Xiufang Ding, Lijie Chen

**Affiliations:** Huzhou Maternity & Child Health Care Hospital, Huzhou 313000, Zhejiang Province, China

## Abstract

In order to improve the quality of life of breast cancer patients, this paper will apply continuous early intervention to the nursing of breast cancer patients. The continuous early intervention nursing model can propose countermeasures for the health problems faced by patients with postoperative chemotherapy. In order to analyze the effect of continuous early intervention nursing on negative emotions and quality of life in breast cancer patients, the effect of continuous early intervention in improving the quality of life of breast cancer patients is analyzed by means of experimental research. The control group is given routine nursing, and the observation group is given continuous early intervention nursing intervention. Moreover, this paper obtains data statistics in combination with statistical analysis. Through the comparison of the test results, it can be seen that the implementation of continuous early intervention nursing intervention in breast cancer patients can improve the nursing effect, effectively relieve the negative emotions of patients, and improve the quality of life of patients.

## 1. Introduction

With the progress of modern medicine and the enhancement of people's awareness of health care, most breast cancer patients can get early diagnosis and early treatment and the long-term survival rate after surgery is also gradually improved. Therefore, how to improve the quality of life of breast cancer patients has attracted widespread attention in the medical community. Quality of life, a multidimensional concept, is people's subjective experience of goals, values, expectations, and living conditions. Clinically, quality of life is commonly used to evaluate the impact of disease and treatment on the physical, psychological, and social functions of patients. The quality of life of breast cancer patients is a dynamic indicator that changes with lifetime and is affected by many factors. Existing studies have shown that patients' physical symptoms, self-esteem, psychological stress, self-efficacy, and ability to cope with and adapt to diseases are all influencing factors of quality of life. First of all, the fact of having breast cancer is a serious stress and crisis event for both the patient and the family members. The diagnosis and surgical treatment of breast cancer is a process that most breast cancer patients have to go through. This process will have a huge impact on the patient's psychological, social, and family functions and then seriously affects the quality of life of breast cancer patients. Secondly, modified radical mastectomy for mastalgia can improve the cure rate of tumors, but it also damages the patient's skin, breast, fascia, muscle, and other tissue structures. This can easily lead to pathophysiological conditions such as soft tissue fibrosis, decreased muscle contractility, disruption of lymphatic pathways, and increased nerve sensitivity. After modified radical mastectomy for breast cancer, the skin lymphedema of the affected limb, the functional impairment of the loyal limb, and the movement disorder of the shoulder joint caused serious distress to the patient and seriously affected the quality of daily life of the patient. Third, the absence of breasts after surgery results in physical defects and changes in women's self-image, resulting in serious damage to the patient's self-esteem. At the same time, changes in self-efficacy and social adaptability affect the patient's normal work and life and reduce the patient's quality of life.

The perioperative period is a dangerous period in terms of the occurrence of negative emotions and abnormal adaptive behavior, which seriously affects the patient's compliance with surgical treatment and greatly affects the patient's prognosis, quality of life, and survival time. The perioperative period is a critical period for the treatment of breast cancer patients, and it is also a period of concentrated outbreaks of various physiological dysfunctions and psychological crises. Studies have shown that breast cancer patients have more psychological problems during the perioperative period and negative emotions such as anxiety are prominent, which is much higher than that of healthy people. However, at the same time, the perioperative period is also a critical period for functional exercise, prevention of complications, psychological adjustment, obtaining more social support, and establishing a good social adaptation function. The early postoperative period of breast cancer is the best time to start functional exercise, which can effectively prevent postoperative upper limb dysfunction. At the same time, family is the most important source of support for perioperative patients. The care, understanding, and support of family members, especially spouses, can enhance the patient's expectation of life, improve self-esteem, effectively enhance the patient's confidence in coping with difficulties, and better maintain their social adaptation function, thereby improving the quality of life of breast cancer patients.

## 2. Related Work

In [1], a survey of 200 breast cancer patients showed that a total of 14 symptoms were significantly negatively correlated with the quality of life of patients. Among them, the top five symptoms were lack of vitality, hair loss, mental stress, sweating, and anxiety. The top 5 most distressing symptoms for patients were hair loss, feeling “I do not look like myself,” poor sleep, loss of appetite, and lack of energy. The research in literature [2] shows that the pain and edema of the affected limb after surgery have a certain degree of influence on the quality of life of loyal patients and the painful mouth maggots will also affect the quality of life of patients. In improving the quality of life of patients, the first thing to do is to maximize the control of symptoms [3]. Medical staff should pay enough attention, because these symptoms will accompany patients through every day; if these symptoms improve, the quality of life of patients will naturally improve. Literature [4] investigated the quality of life of 70 cancer patients before and after cancer pain treatment. The results showed that pain can comprehensively affect the quality of life of patients and effective analgesic treatment can significantly improve the quality of life of patients. Literature [5] systematically evaluated the effect of functional rehabilitation training in patients after breast cancer surgery, and the results showed that progressive limb rehabilitation training and whole body rehabilitation exercise in patients after breast cancer surgery can effectively improve the function of the affected limb and improve the quality of life. Relief of fatigue symptoms in patients with chemotherapy and radiotherapy has a certain effect. Individualized aerobic exercise can improve the patient's fatigue state and improve the patient's quality of life [6]. Postoperative breast cancer patients experience heaviness, swelling, tenderness, and numbness before developing upper extremity lymphedema, so early guidance and intervention are imperative. Clinical nurses should provide patients and their families with personal care guidance for lymphedema, so that patients and their families can master the correct long-term supportive treatment methods for the prevention of lymphedema [7]. Breast cancer patients have more psychological problems in the process of diagnosis, treatment, and rehabilitation, which has been proved by more and more studies [8]. Suffering from cancer is a strong stress stimulus for most people. Breast cancer and its surgical treatment can lead to obvious stress reactions in patients, such as anxiety, depression, anger, fear, and other negative emotions, which affect treatment and recovery. To a certain extent, the quality of life of patients and the whole family decreases [9]. Literature [10] studies have shown that systematic psychological intervention for breast cancer patients can effectively alleviate their negative emotions and improve their quality of life. Literature [11] believes that negative life events, social support, depression, and other psychosocial factors have a greater impact on the immune function of cancer patients. Most breast tumor patients have a strong stress response, and their immune function is significantly inhibited, and the stronger the stress response, the more severely inhibited their immune function. After timely psychological intervention, providing spiritual comfort, support, persuasion, and hints, the patient can quickly control the chaotic thinking and feelings and the psychological response and immune function can be effectively improved. Perioperative breast cancer patients have serious negative emotions, and psychological intervention can significantly improve the treatment of their physical diseases and their quality of life. The results of the study also showed that through psychological intervention, the negative emotions such as anxiety and depression in different cancer patients were significantly reduced and the quality of life was significantly improved. Yang Qiaoju's psychological intervention research confirmed that social psychological factors are closely related to the occurrence and development of malignant tumors, which is why the psychological intervention for patients with malignant tumors received better results. The main reason is that psychological intervention can better relieve some of the patients' psychological pressure and mental burden. It enables patients to receive treatment under a good emotional experience, and at the same time, a healthy psychological condition and a good mood can improve immunity and improve the quality of life through the role of the neuroendocrine immune system, forming a virtuous circle, which further enhances the patient's confidence in treatment. On the other hand, health education before and during chemotherapy enables patients to understand a lot of chemotherapy knowledge, eliminate patients' doubts and worries, help patients establish positive coping strategies, enhance self-care awareness, and actively help them cooperate with treatment. Finally, psychological intervention, such as one-on-one conversation and communication, enables patients to feel the greatest support and care from medical staff and helps patients adjust to problems caused by diagnosis and treatment [12]. The psychological intervention measures used in the study can effectively promote the improvement of the quality of life of patients with breast cancer after chemotherapy and contribute to the overall recovery of the patients. Clinical medical staff should understand the poor psychology of patients undergoing chemotherapy after breast cancer surgery, master the methods of psychological intervention, and actively carry out psychological intervention to improve the quality of life of patients undergoing chemotherapy after breast cancer surgery [13]. The results of literature [14] show that the psychological disorders of postoperative patients are closely related to age. The older they are, the lighter the psychological barrier, because they and their husbands have high hopes for quality of life and prolonging life and have little requirements for sex. The younger the age, the more severe the mental disorder. Improvement can be achieved to a large extent through psychological care. Unilateral mastectomy did not affect the postoperative quality of sexual life. In this process, medical staff's sense of responsibility and psychological communication ability and skills play a leading role. Correct psychological guidance has a significant effect on reducing postoperative sexual dissatisfaction. The main reasons for patients' anxiety and low self-esteem before and after surgery were concerns about affecting their sexual life. It is advised to inform the patient that postmastectomy will not affect the couple's sexual life. However, it should also be noted that the operation will bring inconvenience and embarrassment to the sexual life of the patient and her husband. The patient will be ashamed to expose herself due to physical defects, and at the same time, she will worry that sexual life will have adverse effects on her body. In response to this problem, patients and their husbands should be informed that this deficiency can be compensated by nonphysical love at this stage [15]. After a period of time, the psychology of both parties adapts to this reality and it will naturally get better. Psychological care can help patients adapt to the physical changes caused by mastectomy as soon as possible, influence patients to establish a correct understanding and evaluation of such changes, help them adjust to their psychological state in a timely manner, and help them to be confident in their future life. Psychological counseling and guiding intervention are very important to eliminate the anxiety and inferiority of patients through enlightenment. Psychological intervention can transform the spouse's sexual attitude and improve the quality of sexual life. Therefore, as long as the patients and their families are relieved of their ideological concerns, psychological intervention can reduce the occurrence of postoperative sexual life dissatisfaction [16].

Studies have shown that 30% of breast cancer patients show varying degrees of anxiety and depression and their quality of life is significantly lower than that of the normal population. Although the American Society of Clinical Oncology (ASCO) has developed assessments and measures to manage symptoms such as anxiety and depression in cancer patients, many breast cancer patients undergoing chemotherapy still report a high number of unmet needs, including physical, psychological, and social support and spiritual care [17]. A survey of support needs for breast cancer patients undergoing chemotherapy showed that younger patients had more information needs about the health care system and sexuality and that unmet needs were positively associated with patient symptom distress scores. The results of a survey on the quality of life of long-term breast cancer survivors in literature [18] show that the quality of life of breast cancer survivors is relatively satisfactory, but there are still physical and psychological diseases, and anxiety and depression are related to the reduction of quality of life. Literature [19] shows that the longer the breast cancer chemotherapy patients continue early care, the better their cognition, behavior, and status of the disease and the more confident they are to complete the treatment. During hospitalization, cancer patients can be cared for by medical staff, but their treatment time in the hospital is not long, and most of the patients recuperate at home during the intermittent period of treatment. Corresponding support and guidance are of great significance. Patients are eager to return to normal life after discharge, and they need to be managed to prevent tumor recurrence, symptom control, rehabilitation exercises, etc., to reduce physical and psychological discomfort. Rehabilitation will be of great benefit.

## 3. Materials and Methods

### 3.1. Research Object

In the experiment, breast patients who are admitted to the hospital were selected as the research objects. Inclusion criteria are as follows: female patients, who were conscious and normal, underwent pathological and imaging examinations, met the diagnostic criteria for breast cancer, received chemotherapy after surgery, had complete clinical data, provided informed consent, and obtained approval by the medical ethics committee. Exclusion criteria are as follows: showed poor active cooperation ability during treatment or withdrawal from the study for some reason; had systemic chronic disease or liver and kidney dysfunction; had nonprimary breast cancer; had speech, communication, audio-visual, behavioral, and other obstacles. They are equally divided into the observation group and control group completely by the random number table method. There is no significant difference in general data between the two groups (*P* > 0.05), which is comparable. There is no statistical difference in the age composition and educational level composition of the two groups of patients (*P* > 0.05), which are comparable. This study was approved by the hospital ethics committee.

### 3.2. Experiment Method

When the patients in the two groups are discharged from the hospital after the operation, the responsible nurses provided health guidance for discharge after the modified radical mastectomy for breast cancer. It includes dietary guidance, key points of limb protection, functional exercise of the affected limb, guidance on identifying flap necrosis and subcutaneous effusion, maintenance of drainage tubes, monitoring of drainage fluid, and guidance on taking medicines for discharge. At the same time, the patients on every Monday afternoon (control group) or every Wednesday afternoon (observation group) made an appointment to return to the hospital to observe the wound. One month after the patients are discharged from the hospital, the recovery status of the skin flap and the functional recovery of the upper limb on the affected side were evaluated.

On this basis, the observation group implemented diversified continuous early interventions. (1) 1–3 days before discharge, the patients and their families will be evaluated for their psychosocial status, a personalized continuous early intervention plan will be developed, and hospital contact information will be issued. The specific methods and contents of continuous early intervention are shown in Table 1. (2) Composition and training of successive early intervention teams: The ward has 32 beds and 13 nurses. The continuous early intervention group consisted of 2 deputy chief physicians of breast surgery, 2 nurses in charge, and 5 nurses who had worked for more than 5 years. Among them, there is 1 lymphedema therapist and 1 psychological counselor. The training content includes breast cancer-related disease knowledge, wound management, physical function assessment, common complication assessment and coping strategies, listening and talking skills, guidance education on negative emotions, service awareness, nutrition, etc. (3) Establishment of a patient basic information table: the main contents of the control group information table include the patient's name, hospital number, age, admission date, operation date, discharge date, discharge diagnosis, phone number, diet, sleep, mood, flap recovery, incision suture removal time, amount of drainage fluid, upper limb swelling, and upper limb function recovery. On this basis, the observation group information table adds the follow-up date, follow-up content, and answers to difficult questions. (4) Items of continuous early care.

*(1) Incision Management*. ① It is necessary to observe the color, temperature, and tension of the wound flap to identify flap necrosis and subcutaneous effusion. If it is found that the incision is red and swollen, there is a sense of fluctuation under the skin, or if the color of the skin flap is purple, we should contact the management physician in time and deal with it in time. ② It is necessary to keep the incision dressing clean and dry, and it is advised not to scratch it with the hands to avoid infection.

*(2) Drainage tube management*. ① It is necessary to squeeze the drainage tube correctly to keep the drainage smooth. ② It is necessary to maintain the effective negative pressure suction of the negative pressure drainage bottle. ③ It is necessary to pour the drainage fluid regularly every day. If it is found that the drainage fluid suddenly decreases sharply, combined with chest wall pain or more fluid leakage from the drainage tube orifice, the patient needs to go to the hospital in time. At the same time, patients need to be informed of the dangers of not pouring the drainage fluid in time and the importance of recording the drainage fluid to improve their compliance.

*(3) Process of Functional Exercise of the Affected Limb*. It is necessary to formulate a personalized functional exercise plan for the affected limb for the patient according to the patient's description, postoperative days, and wound healing. At the same time, it is necessary to invite family members to participate in the plan and inform patients and family members of the purpose and significance of functional exercise of the affected limbs, so as to improve patients' compliance and family members' awareness of supervision. 

*(4) Guidance on Diet and Emotional State*. It is necessary to distribute small prescriptions for breast cancer nutrition diets, instruct patients to arrange meals reasonably, and fast from greasy, estrogen-rich foods, or drugs. 

*(5) Psychosocial Support*. It is necessary to assist patients in discovering social support resources around them, so that they can obtain support effectively, encourage family members, especially spouses, to provide psychological support, and maintain emotional stability. At the same time, patients need to be informed that they can consult follow-up staff if they have anxiety, depression, and other emotions or poor sleep. In addition, it is necessary to encourage participation in the activities of the Pink Ribbon Club and the promotion of rehabilitation-themed salons to provide patients with more information and psychological support.

The adverse mood changes of the two groups of patients were recorded. Adverse mood changes were evaluated using the Self-Rating Anxiety Scale (SAS) and Self-Rating Depression Scale (SDS). They are performed before treatment and 3 months after patient care. The scales include 20 items, and the cutoff value is 50 points. The higher the score, the more severe the anxiety or depression. Changes in the quality of life of patients before and after nursing are recorded, and the European Organization for Cancer Treatment and Research is used to develop the RTC-QOL-C30 scoring scale. The higher the functional score, the better the quality of life of the patients. The nursing satisfaction of the two groups of patients is compared using a self-made questionnaire, which is divided into satisfied and dissatisfied levels. Before and after nursing, the health knowledge mastery of the two groups of patients is measured. In this experiment, we design a questionnaire on health knowledge of patients after chemotherapy, including five dimensions, representing the most basic chemotherapy support, skin reaction, and diet. The score adopts a three-level scoring method, and the patient never understands complete mastery of 3 points. The higher the score, the higher the patient's mastery of health knowledge.

## 4. Results

After nursing, the SAS and SDS scores of the two groups are significantly decreased (both *P* < 0.05). There are statistically significant differences in the SAS and SDS scores between the two groups (both *P* < 0.05), as shown in Tables 1 and 2. The corresponding statistical chart is shown in Figure 1 and 2.

After nursing, the quality of life scores of the two groups are improved (both *P* < 0.05). The quality of life scores of the observation group after intervention are significantly better than those of the control group (all *P* < 0.05), as shown in Tables 3–9. The corresponding statistical chart is shown in Figures 3–9.

## 5. Analysis and Discussion

In recent years, the incidence of breast cancer in China has shown a gradually increasing trend and the affected population is getting younger. Statistics show that breast cancer has acquired the third place among all malignant tumors. Although the diagnosis and treatment techniques have been improved, the functional rehabilitation of nurses after surgery will inevitably lead to the loss of hope for many patients. Therefore, it is of great practical significance to study which nursing methods are used to improve patients' negative emotions and quality of life. The adverse reactions of breast cancer patients during treatment not only affect the patients' recovery but also affect their psychological status, resulting in a decline in the patients' quality of life. In the analysis of this group, the focus is on the application of continuous early care in breast cancer. With the rapid development of nursing disciplines, a lot of efforts have been made in the nursing work of breast cancer chemotherapy at home and abroad. Continuous early care is given to implement discharge care on the basis of overall care, to ensure that patients can receive the same care as inpatient care after hospitalization, to effectively ensure the rehabilitation of patients with humerus, and to reduce the case fatality rate of patients. Continuous early care for breast cancer patients can effectively reduce CRF during chemotherapy and improve patient satisfaction. It shows that the implementation of continuous early nursing care for breast cancer patients is helpful for the mastery of patients' health knowledge and has an important effect on improving the relationship between nurses and patients, which is consistent with the results reported in previous studies. Moreover, various adverse reactions after breast cancer treatment seriously affect the quality of life of patients. As patients spend most of their time recovering at home, this prevents continuation of care. The implementation of continuous early care can ensure the continuity and integrity of nursing intervention and, at the same time, can improve the nursing ability of patients themselves and their families and improve the quality of life of patients. Before nursing, there is no significant difference in the SAS score and SDS score between the two groups (*P* < 0.05). After nursing, the SAS and SDS scores of the two groups are significantly decreased (both *P* < 0.05) and the SAS and SDS scores of the observation group are significantly lower than those of the control group at the same time after nursing (both *P* < 0.05). Moreover, the quality of life of the patients in the observation group after intervention is significantly better than those in the control group except for loss of appetite, constipation, diarrhea, economy, and other dimensions (all *P* < 0.05). The research results show that the implementation of continuous early care can improve the role function and emotional function of patients, indicating that the implementation of continuous early care can effectively reduce the adverse symptoms of patients and extend clinical intervention from the hospital to the family.

It is necessary to standardize the way of continuous early care and improve the professional quality of nursing staff. Moreover, continuous early care needs to organically combine the enthusiasm of patients for self-care and the enthusiasm of nurses by carrying out a variety of health education activities, which increases the trust of patients in nursing staff and makes the satisfaction of patients improve. In this study, continuous early care team members were trained once a week on breast cancer specialist knowledge, prevention and countermeasures for common complications after breast cancer surgery, identification of common psychological problems and emotional management, and other related subjects to improve their professional quality. At the same time, relevant guidelines and standards are formulated for the content and operation procedures of continuous early care, to standardize the professional behavior of nursing staff and to improve the quality of continuous early care. At the same time, it is necessary to use a convenient and economical network platform to provide consultation services, implement health guidance, and facilitate the implementation of continuous early care for patients in various places. Through face-to-face guidance and communication, the patients' compliance with treatment and functional rehabilitation of the affected limbs after discharge can be effectively improved and their emotions can be relieved in time. However, the disadvantage is that it is limited by time; through telephone follow-up, patients can feel the humanistic care of the hospital and improve nursing satisfaction. To sum up, continuous early nursing can effectively reduce postoperative complications of breast cancer and promote functional recovery of the upper limbs on the affected side. The establishment of a high-quality continuous early care team is the guarantee of continuous early care. Therefore, we need to develop a personalized continuous early care program and use a variety of continuous early care pathways. For example, carrying out continuous early care by means of appointment follow-up time, setting up QQ group, WeChat group, online consultation and answering questions, follow-up consultation, telephone follow-up, etc., is conducive to achieving good results.

## Figures and Tables

**Figure 1:** Statistical chart of comparison of SAS of patients.

**Figure 2:** Statistical chart of comparison of SDS of patients.

**Figure 3:** Statistical chart of comparison of physical functions.

**Figure 4:** Statistical chart of comparison of role functions.

**Figure 5:** Statistical chart of comparison of emotional functions.

**Figure 6:** Statistical chart of comparison of social functions.

**Figure 7:** Statistical chart of comparison of cognitive functions.

**Figure 8:** Statistical chart of comparison of overall functions.

**Figure 9:** Statistical chart of comparison of nausea and vomiting.

**Table 1:** Comparison of SAS of patients.

Number	Control group	Test group	Number	Control group	Test group
1	42.71	35.35	16	53.08	39.05
2	52.64	41.91	17	56.50	48.48
3	54.83	40.62	18	47.36	40.73
4	45.49	44.22	19	57.99	39.12
5	53.51	35.59	20	58.50	36.87
6	54.95	45.78	21	56.38	43.08
7	56.53	38.86	22	43.46	40.06
8	53.35	36.30	23	57.13	37.50
9	47.60	44.38	24	53.85	34.71
10	51.82	42.15	25	55.27	47.48
11	51.85	35.95	26	52.82	38.31
12	54.46	41.98	27	48.29	34.58
13	57.91	39.14	28	52.59	47.44
14	43.61	47.36	29	49.47	37.11
15	52.22	44.63	30	56.12	38.84

**Table 2:** Comparison of SDS of patients.

Number	Control group	Test group	Number	Control group	Test group
1	48.14	36.17	16	53.55	41.48
2	54.89	40.81	17	44.41	44.10
3	47.03	42.96	18	47.72	38.37
4	41.76	35.70	19	54.18	35.71
5	43.37	34.31	20	48.03	40.14
6	43.33	36.20	21	40.95	35.58
7	52.35	42.92	22	49.46	40.02
8	53.98	44.00	23	54.90	37.15
9	46.87	42.09	24	47.66	33.27
10	48.35	35.37	25	54.51	33.76
11	53.90	38.04	26	52.98	40.77
12	52.16	36.29	27	41.77	38.54
13	46.79	39.43	28	40.45	43.13
14	45.08	37.38	29	50.03	35.72
15	51.38	37.74	30	42.75	36.00

**Table 3:** Comparison of physical functions.

Number	Control group	Test group	Number	Control group	Test group
1	60.22	62.51	16	16	89.80
2	67.52	60.65	17	17	80.71
3	85.66	67.10	18	18	88.88
4	75.84	74.12	19	19	89.17
5	89.19	84.65	20	20	75.13
6	74.98	60.44	21	21	75.65
7	84.85	74.88	22	22	68.21
8	65.66	64.02	23	23	76.10
9	70.70	56.68	24	24	62.12
10	72.31	79.06	25	25	89.54
11	79.44	78.62	26	26	86.62
12	79.27	73.09	27	27	63.12
13	88.72	69.26	28	28	85.95
14	66.41	82.70	29	29	78.77
15	65.72	73.12	30	30	67.66

**Table 4:** Comparison of role functions.

Number	Test group	Control group	Number	Test group	Control group
1	72.51	25.14	16	58.78	20.80
2	42.11	10.61	17	55.06	41.51
3	63.22	23.69	18	84.62	9.58
4	38.19	12.13	19	82.83	67.74
5	60.72	21.27	20	63.07	71.45
6	85.54	10.77	21	62.56	35.48
7	73.24	66.44	22	44.92	12.55
8	55.21	67.04	23	58.52	19.52
9	66.24	64.99	24	62.66	37.47
10	47.34	10.27	25	52.63	57.30
11	75.41	10.98	26	49.80	32.81
12	86.77	16.20	27	42.40	69.36
13	50.82	8.90	28	76.56	44.75
14	40.35	16.97	29	44.35	45.52
15	84.68	35.54	30	56.09	68.39

**Table 5:** Comparison of emotional functions.

Number	Test group	Control group	Number	Test group	Control group
1	73.59	70.26	16	86.55	50.07
2	86.60	61.65	17	58.86	30.22
3	64.98	42.94	18	87.15	60.08
4	64.27	55.82	19	49.14	64.89
5	80.67	59.25	20	68.96	51.92
6	75.90	27.73	21	76.09	43.44
7	69.10	58.39	22	51.02	53.99
8	59.84	57.25	23	76.64	34.23
9	55.37	40.99	24	66.98	55.92
10	59.22	73.88	25	73.31	47.99
11	63.28	33.96	26	47.62	67.64
12	50.06	63.85	27	66.81	28.48
13	85.04	74.15	28	86.94	52.39
14	52.09	46.12	29	75.52	74.05
15	81.02	65.31	30	50.51	38.18

**Table 6:** Comparison of social functions.

Number	Test group	Control group	Number	Test group	Control group
1	77.77	16.88	16	49.94	37.74
2	41.33	23.55	17	78.33	42.01
3	65.44	48.09	18	51.93	13.18
4	30.19	18.93	19	68.79	9.50
5	76.75	53.52	20	41.46	54.55
6	33.90	52.69	21	49.72	53.34
7	55.92	35.04	22	36.42	25.83
8	31.43	39.29	23	72.48	51.37
9	46.87	38.26	24	57.09	56.74
10	47.74	36.09	25	51.37	16.48
11	40.73	35.25	26	53.79	42.50
12	52.18	41.80	27	42.09	21.45
13	49.85	53.99	28	43.54	10.56
14	37.80	49.83	29	34.89	44.72
15	59.40	22.96	30	68.69	39.99

**Table 7:** Comparison of cognitive functions.

Number	Test group	Control group	Number	Test group	Control group
1	90.34	89.35	16	89.60	74.65
2	80.79	82.24	17	97.91	84.85
3	84.33	55.42	18	70.67	64.41
4	81.20	87.95	19	79.90	79.35
5	72.15	94.52	20	67.34	83.56
6	69.23	93.60	21	67.91	83.40
7	69.16	83.73	22	85.52	55.87
8	88.36	62.65	23	89.13	88.35
9	90.19	78.73	24	89.55	91.59
10	95.94	62.32	25	72.36	58.24
11	74.94	83.89	26	94.34	78.49
12	73.20	53.63	27	68.27	88.63
13	77.61	69.02	28	70.09	57.36
14	79.42	60.01	29	94.04	92.74
15	92.74	80.68	30	95.80	52.62

**Table 8:** Comparison of overall functions.

Number	Test group	Control group	Number	Test group	Control group
1	31.64	53.99	16	42.71	23.39
2	24.70	23.35	17	59.09	54.13
3	68.43	31.32	18	71.18	35.44
4	73.46	36.03	19	33.71	43.98
5	62.70	23.88	20	33.07	41.21
6	25.57	35.05	21	20.95	48.32
7	39.83	28.19	22	61.42	29.16
8	69.83	38.27	23	24.72	23.74
9	40.12	23.99	24	70.87	38.72
10	47.08	32.65	25	58.63	21.97
11	42.73	30.57	26	48.09	22.39
12	25.31	50.02	27	49.42	44.41
13	56.77	38.41	28	32.59	43.38
14	28.58	50.82	29	67.90	31.31
15	60.00	45.00	30	56.40	38.79

**Table 9:** Comparison of nausea and vomiting.

Number	Test group	Control group	Number	Test group	Control group
1	71.95	96.44	16	67.51	87.69
2	83.21	75.07	17	46.71	64.25
3	71.57	94.08	18	82.57	91.64
4	43.23	62.72	19	77.94	75.06
5	71.94	64.00	20	50.80	64.78
6	75.31	93.38	21	55.16	71.32
7	89.72	61.94	22	46.77	67.39
8	59.10	86.00	23	50.23	66.08
9	82.30	68.92	24	94.41	83.64
10	41.97	65.84	25	68.52	63.21
11	71.04	85.39	26	95.22	74.30
12	71.35	73.55	27	95.94	73.18
13	57.62	78.71	28	93.88	65.43
14	73.52	75.45	29	80.60	66.22
15	76.92	65.44	30	73.32	94.98

## Data Availability

The labeled datasets used to support the findings of this study are available from the corresponding author upon request.
